The article "Application of Adaptive Neural Network Algorithm Model in English Text Analysis" was retracted in 2023. Reasons: signs of a paper mill; suspected computer-generated content; unreliable results or conclusions; concerns about the data.

# Application of Adaptive Neural Network Algorithm Model in English Text Analysis

**DOI:** 10.1155/2022/4866531

**Published:** 2022-05-26

**Authors:** Maosheng Hung, Meijin Hsiao

**Affiliations:** ^1^School of Foreign Languages, Fuzhou University of International Studies and Trade, Fuzhou, Fujian 350202, China; ^2^School of Art and Design, Fuzhou University of International Studies and Trade, Fuzhou, Fujian 350202, China

## Abstract

Based on the existing optimization neural network algorithm, this paper introduces a simple and computationally efficient adaptive mechanism (adaptive exponential decay rate). By applying the adaptive mechanism to the Adadelta algorithm, it can be seen that AEDR-Adadelta acquires the learning rate dynamically and adaptively. At the same time, by proposing an adaptive exponential decay rate, the number and method of configuring hyperparameters can be reduced, and different learning rates can be effectively obtained for different parameters. The model is based on the encoder-decoder structure and adopts a dual-encoder structure. The transformer encoder is used to extract the context information of the sentence; the Bi-GRU encoder is used to extract the information of the source sentence; and the gated structure is used at the decoder side. The input information is integrated, and each part is matched with different attention mechanisms, which improves the model's ability to extract and analyze relevant features in sentences. In order to accurately capture the coherence features in English texts, an improved subgraph matching algorithm is used to mine frequently occurring subgraph patterns in sentence semantic graphs, which are used to simulate the unique coherence patterns in English texts, and then analyze the overall coherence of English texts. According to the frequency of occurrence of different subgraph patterns in the sentence semantic graph, the subgraphs are filtered to generate frequent subgraph sets, and the subgraph frequency of each frequent subgraph is calculated separately. The overall coherence quality of English text is quantitatively analyzed by extracting the distribution characteristics of frequent subgraphs and the semantic values of subgraphs in the sentence semantic graph. According to the experimental results, the algorithm using the adaptive mechanism can reduce the error of the training set and the test set, improve the classification accuracy to a certain extent, and has a faster convergence speed and better text generalization ability. The semantic coherence diagnosis model of English text in this paper performs well in various tasks and has a good effect on improving the automatic correction system of English composition and providing reference for English teachers' composition correction.

The article "Application of Adaptive Neural Network Algorithm Model in English Text Analysis" was retracted in 2023. Reasons: signs of a paper mill; suspected computer-generated content; unreliable results or conclusions; concerns about the data.

## 1. Introduction

Eighty percent of the web pages or information on the Internet are in English, and various English texts (such as news, reviews, and emails) are filled with all aspects of people's life and work [1]. Therefore, the research on new English text semantic feature extraction and its understanding methods will not only help further solve a series of key problems in the field of artificial intelligence such as current text classification, machine translation, automatic question answering, text generation, and human-computer interaction but also help facilitate communication and understanding between different languages [2]. At the same time, with the maturity of key technologies of artificial intelligence such as natural language processing, automated semantic understanding of English texts can quickly understand the international situation, grasp the direction of international public opinion, and protect national information security [3, 4]. Therefore, with the advancement of natural language processing in the direction of natural language understanding, solving the hot and difficult problems of text semantic feature extraction and semantic understanding methods in natural language understanding will definitely play an important role in the development of natural language understanding research [5].

In recent years, with the rapid development of neural networks, especially the emergence of deep learning technology that relies on large-scale data training methods, major breakthroughs have been made in natural language processing, which has led to a new dawn and direction for machine understanding of text [6]. Bengio first proposed that the use of deep neural networks to build pretrained language models can learn semantic information in text data. On this basis, the word vector model of distributed representation has achieved great success. At present, researches on obtaining text representations relying on pretrained language models emerge in an endless stream [7]. Among them, Google's Bidirectional Encoder Representations from Transformers (BERT) model trains language models by masking some words in the text [8]. This automatic noise encoding method obtains text semantic representation and achieves better results in downstream natural language processing tasks, especially in reading comprehension tasks. Subsequently, Carnegie Mellon University and Google Brain launched the XLNet model, an autoregressive attention model that can obtain richer contextual information. It is obviously unrealistic to rely on humans to analyze, understand, and classify these massive texts. However, text understanding is the most critical technology for machines to ultimately realize intelligence. Therefore, in many artificial intelligence application scenarios, the study of computer understanding of the text is of crucial significance.

The article "Application of Adaptive Neural Network Algorithm Model in English Text Analysis" was retracted in 2023. Reasons: signs of a paper mill; suspected computer-generated content; unreliable results or conclusions; concerns about the data.

For the learning rate, this paper proposes an adaptive mechanism and applies the adaptive mechanism to the Adadelta algorithm. We use this algorithm to optimize the weight distribution of LSTM and LeNet. This paper presents the design and methodology of each part of the English text analysis model. The overall structure of the automatic grammatical error correction model is given, and the preprocessing methods of the model are introduced, including the data augmentation method based on fluency and the dynamic word vector representation method. After that, the encoder module is introduced, which mainly includes two parts, namely the context information encoder and the Bi-GRU encoder. The masking method in the decoder and the specific details of the gating structure are introduced. The decoding strategy of the encoder-decoder structure is given, including an overview of existing decoding algorithms and the dynamic beam search method proposed in this paper. This paper expounds on the corpus used in the model and some evaluation criteria of the model. Finally, the experiments performed by this model are expounded, which are the subgraph screening experiment, the incoherent sentence extraction experiment, the sentence sorting experiment, and the comparison experiment with the teacher's score, and the results of the experiment are analyzed in detail.

### 1.1. Related Work

Scholars summarized and established the framework of the statistical language model on the basis of N-gram (N-gram) and called it a neural network language model (NNLM) [9]. The NNLM uses the nonlinear output function of the neural network to extract text. The semantic features of the word vector provide the cornerstone for the subsequent research on the word vector Word2Vec semantic feature representation model.

The success of the NNLM is that it solves two problems. One is that in the statistical language model, we need to calculate the probability distribution of a word under the current text conditions; the other is the expression problem of word vectors concerned in the vector space model, that is, the problem of text representation. By introducing a continuous word vector assumption and a smooth probability distribution model and by modeling the probability distribution of words in a text sequence in a continuous space, the word vector expression and probability distribution of words are obtained at the same time. This is also because the continuous vector representation method can alleviate the problem of data sparseness to a certain extent.

The article "Application of Adaptive Neural Network Algorithm Model in English Text Analysis" was retracted in 2023. Reasons: signs of a paper mill; suspected computer-generated content; unreliable results or conclusions; concerns about the data.

Despite the success of the NNLM in a text representation, NNLM also suffers from several problems [10]. First of all, the NNLM can deal with sequence problems, but the ability to deal with sequences is not strong. When the sequence length exceeds 10, the number of model parameters is huge and brings greater computational pressure. In Bengio's paper, they increased the sequence length. Although this is a great improvement over the binary and ternary grammar models, the model still lacks flexibility. Second, due to the huge amount of computation, the NNLM takes a long time to train, which seriously affects its practicability. In order to solve these problems, scholars modified the NNLM and proposed the word vector Word2Vec model [11, 12].

Text understanding methods based on the semantic network usually obtain the semantic similarity or correlation between words by calculating the semantic similarity between words [13]. It should be pointed out that similarity and relatedness are not the same concept. Semantic similarity means that two words have similar meanings, or the concepts they represent have similar characteristics. For example, “Microsoft” and “Google” have similar semantics, both being tech companies. The words “car” and “journey” are not semantically similar, but these two words are related, and both are related to transportation [14, 15].

The BERT model is mainly implemented through sentence-level negative sampling, specifically, the task of predicting whether a sentence is a continuous text. First, given a sentence, its next correct sentence is regarded as a positive example, and a sentence is randomly sampled as a negative example, and then the classification task is performed at the sentence level. At the same time, the biggest contribution of BERT is to transfer a large number of traditional downstream specific tasks to pretrained word vectors. The text word vectors obtained in this way and simple fine-tuning can meet most tasks; of course, this is based on the huge amount of data and parameter support.

Pretraining methods usually build text-related semantic information on the basis of training language models and then design different evaluation indicators for text understanding according to different tasks. Generally, text understanding methods based on pretrained language models require large-scale data as support [16]. Text understanding methods based on external knowledge mainly provide relevant information for text understanding through existing knowledge bases, but such methods require manual annotation of knowledge base resources as a comparison of semantic similarity. At the same time, such methods also need to be better at incorporating background knowledge into the representation model [17–19].

The article "Application of Adaptive Neural Network Algorithm Model in English Text Analysis" was retracted in 2023. Reasons: signs of a paper mill; suspected computer-generated content; unreliable results or conclusions; concerns about the data.

Relevant scholars strengthen the model's judgment and reasoning on common sense problems by introducing the common sense information of ConceptNet into the text understanding model [20, 21]. Specifically, for each sample, first, it is necessary to find out the multi-hop paths related to it in the knowledge base, and the entities contained in it appear in the question or document of the sample. Finally, some paths with the highest scores are picked from the output generated by all paths, which are external common sense information that may be helpful to the sample [22, 23].

## 2. Methods

### 2.1. Adaptive Mechanism

Choosing an appropriate learning rate for stochastic gradient descent (SGD) can be very difficult. A learning rate that is too small will lead to a slow convergence rate, while a learning rate that is too large will hinder the convergence rate, which may cause the loss function value to oscillate around the optimal value and may even cause divergence. In addition, many algorithms based on stochastic gradient descent algorithms with regard to the improvement of the learning rate retain many more sensitive hyperparameters that need to be manually configured. The learning stability of the algorithm depends on the choice of hyperparameters, and there are endless ways to configure the hyperparameters of the learning algorithm. Therefore, it needs to deal with sensitive hyperparameters and go through a manual tuning stage to get the expected performance, and this tuning is very expensive, requiring not only time resources but also human resources; each setup is usually done multiple times in multiple stages of test. Therefore, some approaches are taken in this paper to reduce the total number of hyperparameters.

In this paper, we propose an adaptive exponential decay rate based on the stochastic gradient descent algorithm, using the adaptive exponential decay rate to estimate the first-order moment estimates of the gradient and the noncentral gradient variance (second-order original moment estimates) online. The memory size of our adaptive mechanism (i.e., the size of the exponential decay rate) is similar to the cellular mechanism in long short-term memory (LSTM).

LSTM has an input gate and a forget gate. The input gate controls the flow of new incoming information, and the forget gate is used to retain the previous old information. Our adaptive mechanism is similar to the function of the input gate and forget gate in LSTM and proposes an adaptive exponential decay rate to adapt to the change of the gradient, replacing a part of the historical gradient value with a part of the gradient value of the current step. The difference is that when the current step size is relatively large, the gradient ratio of the current step is expected to be larger. When the current step size is relatively small, it is hoped that the gradient of the current step accounts for a small proportion.

The article "Application of Adaptive Neural Network Algorithm Model in English Text Analysis" was retracted in 2023. Reasons: signs of a paper mill; suspected computer-generated content; unreliable results or conclusions; concerns about the data.

At the same time, the exponential decay rate is adaptively obtained, that is, when the step size taken is larger, the size of the memory of the adaptive mechanism increases. If a smaller step size is taken (increment is 1), the size of the memory of the adaptive mechanism is reduced, that is, when the step size taken is larger, the size of the gradient memory is expected to be larger. When the step size taken is small, the size of the gradient memory is expected to be small. This adaptive exponential decay rate adaptation mechanism enables us to eliminate the sensitive hyperparameter.

Assuming that *m*_*t*_ and *v*_*t*_ are the exponential moving average gradient and the partial variance gradient, respectively, they can also be considered as the first and second moment estimates of the gradient. *β*_*t*_ is the adaptive exponential decay rate at step *t*, and the initial value of the adaptive exponential decay rate is *β*_*0*_ = 0. The first and second moment estimates of the gradient of the adaptive mechanism are calculated as follows:

(1) $$\begin{array}{c} m_{t+1}=\left(1-\beta_{t}\right)g_{t}-2\left|\beta_{t}\right|m_{t-1},\\ v_{t+1}=2\left(1-\beta_{t}\right)g_{t}-\left|\beta_{t}\right|v_{t-1}. \end{array}$$

We expect that the exponential decay rate online estimates of the first-order gradient (moment estimates) and the noncentral variance gradients (second-order original moment estimates) increase when the step size is larger. If the step size taken is smaller (increment is 1), the exponential decay rate is the online estimated first-order gradient (moment estimation), and the noncentral variance gradient (second-order original moment estimation) is reduced, resulting in an adaptive exponential decay rate. That is, when the step size taken is large, it is hoped that the exponential decay rate of the gradient of the current step and the squared gradient of the current step are relatively large; otherwise, when the step size taken is small, it is hoped that the exponential decay rate of all gradients and the squared gradient of the current step is relatively large. The decay rates are all reduced, and the exponential decay rate is dynamically adjusted. Therefore, the adaptive exponential decay rate *β* is designed as follows:

(2) $$\begin{array}{c} \beta_{t}=1-m_{t}\tau_{t}^{-1},\\ \tau_{t}=1-\frac{v_{t}}{1-m_{t}}\tau_{t-1}. \end{array}$$

The article "Application of Adaptive Neural Network Algorithm Model in English Text Analysis" was retracted in 2023. Reasons: signs of a paper mill; suspected computer-generated content; unreliable results or conclusions; concerns about the data.

### 2.2. Overall Design of Adaptive Neural Network Algorithm Model

In the encoder-decoder structure, the encoder mainly represents the input word sequence as an intermediate semantic vector *C*. In the decoder, the intermediate semantic vector *C* is used as input, and the word at the current moment is predicted based on its own generated sequence at the previous moment. The feature of this structure is that it can flexibly handle input and output sequences of unequal lengths, so this model is based on the encoder-decoder structure of the transformer model to design an English text analysis model.

First, the input English text is preprocessed; the training data is mainly expanded; and the first and last labels are added. Then, the amplified parallel sentence pairs are obtained through the ALBERT preprocessing model to obtain the vectorized representation of the sentence, which contains the sentence's part of speech, semantics, and other information. A series of candidate outputs are obtained, and finally, the candidate sentences are screened through the improved beam search algorithm, and the final error correction result is obtained. The overall structure of the English text analysis model is shown in Figure 1.

### 2.3. Preprocessing Method of the Model

More pseudo-parallel sentence pairs are formed by a fluency-based data augmentation method. Sentence fluency is usually measured by sentences written by native English speakers, that is, sentences written by native English speakers are considered fluent. The fluency of a sentence can be calculated by the language model, as shown in the following formula:

(3) $$\begin{array}{c} f\left(x\right)={\left(1-H\left(x-1\right)\right)}^{-1},\\ H\left(x\right)=\frac{1}{x}\prod_{i=0}^{x-1}\log\;P\left(x_{i}|x\geq i-1\right). \end{array}$$

The fluency of the sentence is obtained according to the language model, and the fluency of the reference sentence is used as the standard, and candidate sentences with a score of more than 80% are selected to form parallel sentence pairs with the standard reference sentence and together with the original sentence pairs are used as the training corpus.

In English text, the same word may have different meanings in different contexts. The dynamic word vector technology is to fuse the context information of the word when generating the vectorized representation of the word, so as to obtain different word vector representations according to different contexts. For example, ELMo, BERT, and other models can dynamically represent word vectors according to the word context. However, compared with the over 100M parameters in the BERT base model, the ALBERT base reduces the number of parameters to 12M through cross-layer parameter sharing, embedded parameter factorization, and other methods and achieves results that are very close to the BERT model on SQuAD 2.0. Therefore, in this model, we use the NUCLE corpus to train the ALBERT model and then initialize the input sentence to obtain the word vector.

The article "Application of Adaptive Neural Network Algorithm Model in English Text Analysis" was retracted in 2023. Reasons: signs of a paper mill; suspected computer-generated content; unreliable results or conclusions; concerns about the data.

### 2.4. Context Information Coding Method

The context information encoder (context-before encoder) adopts the structure of the transformer encoding side. There are two reasons for adopting this structure:

1. The long-distance dependency problem has always been a major problem in the processing of long difficult sentences. This problem first appeared in the N-gram model in statistical methods, and it is almost impossible to cover the semantic information of the whole sentence with a fixed-size (usually 3–5 token) window. Later, with the emergence of neural network models such as LSTM and GRU, the long-distance dependency problem has been alleviated to a certain extent, but it is still powerless when dealing with particularly long sentences. During the calculation, the transformer reduces the distance calculation between any two positions of the sentence to a constant through the attention mechanism, which perfectly solves the problem of long-distance dependence.
2. Whether parallel computing can determine the efficiency of model training and affect the effect of the model. The traditional RNN model adopts a sequential calculation method. Each moment depends on the output results of the previous moment. The fully connected network is used between the hidden layers, so it does not have the ability of parallel computing. It is worth mentioning that some scholars have tried to modify the structure of the hidden layer of RNN, such as partially breaking the full connection between the hidden layers according to a fixed time step. Increasing the depth of the network to obtain features at a longer distance achieves a certain degree of parallel computing power, but the actual speed is still not as good as the CNN model. Although CNN can be calculated in parallel, for information transfer over long distances, multi-layer convolution is required to expand the receptive field, and the transformer only needs to perform one calculation.

Combining the above two points, this model will build a context information encoder based on the encoder part of the transformer, and the input selects the first three sentences of the sentence being decoded in the decoder. This is because the original intention of this model design is for Chinese students. The English composition is grammatically corrected, and a composition is usually written based on a theme. Unlike the parallel sentence pairs used in training, the sentences in the composition are related to each other. If you only correct errors based on a single sentence, misjudgment may occur.

The article "Application of Adaptive Neural Network Algorithm Model in English Text Analysis" was retracted in 2023. Reasons: signs of a paper mill; suspected computer-generated content; unreliable results or conclusions; concerns about the data.

For ease of understanding, we use *x* to represent each token in sentence *S*. After vectorizing the input sentence, we can get the first hidden layer state *h*_*0*_ of the model:

(4) $$\begin{array}{c} h_{0}=\left(p-1\right)W_{p}-\beta_{t}W_{c}+\left(q-2\right)W_{Q}, \end{array}$$

where *W*_*c*_ is the word vector embedding matrix, which is used to convert the input token into a word vector; *W*_*p*_ is the position vector embedding matrix, *p* is the position encoding, which is used to provide the position information of the word for the nonsequential encoder; and *W*_*Q*_ is the segment embedding matrix, *Q* is the segment code used to distinguish source and target sequences. In this model, a two-layer context information encoder structure is adopted.

### 2.5. Decoding Design

When processing English text, in addition to the long-distance dependency problem, it is also necessary to solve the variable-length output problem, that is, the length of the input sequence and the length of the output sequence may not be equal. The sequence-to-sequence model, or encoder-decoder structure, can handle the problem of variable-length sequences very well.

In the Masked Multi-Head Attention module of the decoder, the original mask method in the transformer is used as the casual mask because, in the language model, the *i*-th word only depends on the first *i*–1 words, and the position *i* can be hidden through the casual mask, so as to ensure that the prediction will not affect the training effect because of seeing the “future” information. A graphical depiction of the casual mask is shown in Figure 2. The input information is divided into two categories according to the color. The white part represents the historical context information above, which can be “seen” by the decoder, and the red part represents the context information below, which cannot be “seen” by the decoder.

When decoding the source sentence, in order to effectively utilize the coding information of the context, a gating structure is added to integrate the weight of the context attention and the source sentence attention. The calculation steps in the model are described below in combination with the formula. Considering the two parts of Masked Multi-Head Attention and Add and Norm in the decoder as a whole, the output *Y*_*t*_ of this part at time *t* depends on the output *G*_*t*–1_ of the decoder at the first *t*–1 time:

(5) $$\begin{array}{c} Y_{t}=\text{Layer Norm}\left[\text{Multi Head}\left(G_{t-1}\right)-\tau_{t-1}•G_{t-1}\right]. \end{array}$$

After the gating unit, the final output *G*_*t*_ of the decoder is obtained as follows:

(6) $$\begin{array}{c} G_{t}=\tau_{t}Y_{t}+\beta_{t}C_{t}+\left(p-1\right)G_{t-1}. \end{array}$$

The article "Application of Adaptive Neural Network Algorithm Model in English Text Analysis" was retracted in 2023. Reasons: signs of a paper mill; suspected computer-generated content; unreliable results or conclusions; concerns about the data.

### 2.6. Decoding Strategy

After the decoder generates the final probability distribution, it can correspondingly obtain the probability of each word in the vocabulary at the current moment, select the output at the current moment according to the output probability, and adopt a certain decoding strategy. The output of each moment in the decoder is used as the input of the next moment, so the choice of decoding strategy is very important, which directly affects whether the output results of all subsequent moments are accurate.

Beam Search is essentially the idea of the greedy algorithm, but it is improved on its basis, and the candidate search space is expanded by specifying a hyperparameter *K*, which is also called beamwidth. The beam search process retains the *K* candidates with the highest scores at each time step, then at the *k*–1-th time step, the *K* candidates with the highest scores are retained from the *k*–1 candidates. The following formula is used to calculate the score of the candidate queue composed of candidate words:

(7) $$\begin{array}{c} S\left(Y_{t-1}|x\right)=\prod_{i=0}^{t-1}{\left(1-\beta \right)}_{t}•\;\log\;P\left(y_{i}|y_{i-1},x\right). \end{array}$$

The beam search algorithm is a heuristic graph search algorithm that explores the graph by expanding the best nodes in a limited set, keeping only the most promising nodes, and pruning out poor quality nodes. The smaller the beamwidth, the more nodes are pruned, which can improve time efficiency and reduce space consumption when the solution space of the graph is relatively large. However, beam search is to expand the best candidate node by the scores of all the previous words, which leads to an excessive proportion of the parent node. When we expand the last *K* nodes, we will find that the subsequent nodes of the first best node outperform the successor of all other nodes; this parental advantage accumulates as it expands, resulting in the final candidate signal being generated primarily from a single beam, with minor changes in the tail.

There are various improvements to the Beam Search algorithm, such as random sampling and top-k sampling. In random sampling, only the word with the highest probability is selected, but random sampling is performed according to the probability distribution *p* of the words in the dictionary. The advantage of this is to add more randomness, but there will be inconsistencies. In the case of short output, such as chat robots, it cannot meet the needs of high-precision and long text for grammar error correction tasks. In random sampling, there is a hyperparameter *T* (temperature) used to control the probability distribution of the output, as shown in the following formula:

(8) $$\begin{array}{c} p_{i}=\frac{\left(\log\;y_{i}-\log\;T\right)}{\left(\prod \exp\left(y_{i}/T\right)\right)}. \end{array}$$

The larger the value of *T*, the more average the probability distribution, and the greater the randomness of the sampling results; the smaller the value of *T*, the more concentrated the probability distribution, the smaller the randomness during sampling, and the easier it is to get the word with the highest probability.

The article "Application of Adaptive Neural Network Algorithm Model in English Text Analysis" was retracted in 2023. Reasons: signs of a paper mill; suspected computer-generated content; unreliable results or conclusions; concerns about the data.

Top-k sampling only takes the top-*k* words with the highest probability to form a new set and normalizes the probability to obtain a new probability distribution and then sample from the new probability distribution. The downside of this is that a suitable value of *k* is not easy to determine. Because the probability distribution obtained each time is different, it is not possible to obtain the optimal solution in all cases with a constant value of *k*.

## 3. Results and Analysis

### 3.1. Experimental Results of Algorithm Model Analysis

Dropout is to temporarily drop some units in the neural network unit from the network according to a specific probability for the neural network unit during the training process of the deep learning network. Because the algorithm for optimizing the network is generally an optimization algorithm based on the stochastic gradient descent algorithm and because the optimization algorithm based on the stochastic gradient descent algorithm uses random sampling and discarding, each random and mini-batch data (mini-batch) uses a different network. The core point of the dropout technique is to randomly remove certain units and the connections between them from the neural network during training to avoid overfitting between units. During training, samples are sampled from exponentially differenced samples of different “thin” networks; during testing, dropout approximately averages the predictions of these sparse networks, using only a single network for the connected part, making it less weighted. We preprocess each review and tweet data of the English text data set as bag-of-words (BOW), a highly sparse feature vector. We employ a random regularization method (50% dropout noise is used in this paper) to prevent overfitting, and due to its simplicity, it is often used for the bag-of-bag feature during training.

The article "Application of Adaptive Neural Network Algorithm Model in English Text Analysis" was retracted in 2023. Reasons: signs of a paper mill; suspected computer-generated content; unreliable results or conclusions; concerns about the data.

Figure 3 compares the performance of Adadelta, Adam, and Adaptive Neural Network algorithms with and without dropout. It can be seen that when the model uses the dropout technique, the test classification accuracy of all algorithms is relatively high, and the error value is small. Dropout is a useful technique that can improve the performance of neural networks and can be used to prevent overfitting during training. We compare the effectiveness of our algorithm compared to other algorithms by using dropout noise on LSTM networks.

### 3.2. Experiment and Analysis of Subgraph Screening

We employ an improved VF2 subgraph matching algorithm to mine frequently occurring subgraph patterns in the sentence semantic graph and generate our frequent subgraph set through a large amount of training set text. The purpose of mining frequent subgraphs is to capture the unique coherence patterns in the text and use the distribution difference of frequent subgraphs to distinguish texts with good coherence from those with poor coherence. However, there are some frequent subgraphs in the generated frequent subgraphs. In order to verify whether these subgraphs can effectively capture the coherence of text, this paper designs the following experiments to filter frequent subgraphs. This paper selects 500 English compositions with a coherence score between 11 and 15 (total score of 15) from the English learner corpus CLEC as our coherent test sample and 500 English compositions with a score of 7–10. The English compositions between them serve as our less coherent test sample, totaling 400 English compositions. And the number of sentences in these English compositions is not much different. We further filter the frequent subatlas by counting the performance of different frequent subgraphs in the two types of test texts.

According to Figure 4, we can know that most of the frequent subgraphs appear in the two types of test texts with relatively large differences in frequency, which can distinguish texts with good coherence and texts with poor coherence. However, not all frequent subgraph styles can capture the coherence information of the text well. The difference in the average of times is not large, and it cannot capture the coherent pattern of the text very well. If they are placed in the frequent subgraphs, it will affect the frequency distribution of the frequent subgraphs, so we filter such subgraphs. Using this method, we further filter all frequent subgraphs mined by the VF2 algorithm, and finally, we get frequent subgraphs that can effectively capture the coherent patterns in the text. The subsequent experiments also show that the filtered frequent subatlas is more effective.

The article "Application of Adaptive Neural Network Algorithm Model in English Text Analysis" was retracted in 2023. Reasons: signs of a paper mill; suspected computer-generated content; unreliable results or conclusions; concerns about the data.

### 3.3. Experiments and Analysis of Extracting Incoherent Sentences

For the evaluation of the coherence model, a very important point is whether it can identify incoherent sentences. In order to verify the accuracy of the semantic coherence model of this paper in extracting incoherent sentences, relevant experiments were carried out. The corpus used in the experiment is the English learner corpus. A total of 1,000 articles were randomly selected from the corpus as the test set, and 4 incoherent English sentences were randomly inserted into each article as manual annotation of incoherent sentences. When extracting incoherent sentences, this model extracts the entity information and semantic similarity information between sentences and sets an extraction threshold when extracting. Therefore, this paper uses the test set to conduct experiments under different incoherent sentence extraction thresholds to find the most suitable extraction threshold.  Figure 5 shows the results of experiments on incoherent sentence extraction under different thresholds.

In order to verify the performance of the model in extracting incoherent sentences under different numbers of compositions, this paper randomly selects English compositions from the test set and conducts a total of incoherent sentence extraction experiments. The extracted incoherent sentences are compared with the artificially marked incoherent sentences to verify the accuracy of the model in this paper. The experimental results are shown in Figure 6.

From the experimental results in Figure 6, we can see that when different numbers of English compositions are used as test sets, the performance of the model in this paper for extracting incoherent sentences is still relatively stable, and the accuracy of extracting incoherent sentences also varies with the number of compositions. Therefore, the sentence semantic graph model constructed in this paper combines entity word information and semantic similarity information between sentences to extract incoherent sentences in English composition, and it performs well in experiments.

### 3.4. Experiments and Analysis of Sentence Ordering

The sentence ranking task is one of the most commonly used methods to detect coherence analysis models, and it is mainly divided into two types: recognition task and insertion task. The recognition task is to compare an article with an article generated by a random arrangement of its sentences and check whether the model can accurately identify the original article. The insertion task is to compare the original article with a random sentence position transformed article. In this paper, we use the recognition task to test the performance of the model. We randomly selected 100 articles in the COLEN corpus as our test set and shuffled the sentence order in each article to generate 10 shuffled articles. We compare the semantic similarity graph model, entity graph model, and our model on this test set. The real-time performance of sentence ranking of different models is shown in Figure 7.

The article "Application of Adaptive Neural Network Algorithm Model in English Text Analysis" was retracted in 2023. Reasons: signs of a paper mill; suspected computer-generated content; unreliable results or conclusions; concerns about the data.

In the test sample, the sentences of the two articles are the same, but the order of the sentences is different. Identifying the original article requires the model to have a good ability to distinguish coherence. The performance of the entity graph model in the recognition task is not very good. The main reason is that in the test sample, the entity words in the sentence are the same, only the order of the sentences is different, and the entity graph model can only be determined by the distance between the sentences. The edges between sentences are distinguished by different weights, and finally, the average out-degree is calculated to represent the coherence of the text. However, this method can only analyze the coherence in a superficial manner, and its ability to capture the coherence of the text is limited. In comparison, semantic similarity graph models perform better in recognition tasks. This is mainly because it takes into account the semantic information and distance between sentences, but it still uses the feature of average out-degree to represent the text coherence, and the model in this paper combines the entity graph model and the semantic similarity graph model. It uses more complex frequent subgraph frequency and subgraph semantic value features to analyze the coherence of the text, and the accuracy has been improved to a certain extent, which shows that the model in this paper is more able to distinguish the coherence of different texts.

### 3.5. Comparison of Model and Teacher Rating

In order to test the effectiveness of this model in practical use, we apply the model in this paper to correct students' English compositions and compare the results of the corrections with the results of human teachers' scoring. First, we selected 500 student essays from the TECCL corpus as our test set and then invited 5 English teachers to rate the coherence quality of the English essays in the test set. When scoring, only the coherence of the English essays was considered. The score is 25 points, and then we use the English teacher's coherent average score for each composition as the manual score for this composition. Finally, we compare the English composition scoring results of this model with the teacher's manual scoring results to analyze the practical application of the model in this paper. The comparison results of English composition coherence quality scores are shown in Figure 8.

The article "Application of Adaptive Neural Network Algorithm Model in English Text Analysis" was retracted in 2023. Reasons: signs of a paper mill; suspected computer-generated content; unreliable results or conclusions; concerns about the data.

On the whole, the score of the English composition model in this paper is relatively similar to the teacher's manual score for English composition, although there are also some scoring points with a relatively large gap between the two. However, considering the coherent quality correction of English composition, it is a relatively subjective process and is easily affected by various subjective factors. For example, there are too many wrong words in the composition that affect reading; teachers' understanding of the degree of coherence is different; and different teachers' corrections are different. These situations cannot be ruled out manually. Although we use averaging to balance this error, the effect is ultimately limited. Therefore, it is understandable that these scoring points with large gaps appear. However, the correction results of the model in this paper are not much different from the manual correction results, and its correction results in English composition correction are credible.

## 4. Conclusion

This paper proposes an adaptive learning rate to optimize the neural network and reduce the number of hyperparameters. The idea and algorithm process of the adaptive learning rate optimization algorithm are introduced. It mainly introduces a simple and computationally efficient adaptive mechanism based on the existing research. By applying the adaptive mechanism to Adadelta, it can be seen that AEDR-Adadelta dynamically adaptively learns and adjusts parameters while reducing the method of configuring hyperparameters by adjusting only one hyperparameter and effectively assigning different learning rates to different parameters. We design and implement an automatic grammar error correction model that can extract historical sentence information as a reference. The overall model is based on the encoder-decoder framework, and the historical sentence information and the current sentence information are extracted through two different encoder structures. We combine the attention mechanism to integrate the information of the two parts in the decoder and output the final predicted sentence. After representing the text as a sentence semantic graph, we analyze the overall coherence of the text by analyzing the features of the graph. Different from the central measure of the average out-degree in the entity graph, which reflects the overall coherence of the English text, in this model, we pay more attention to the connection mode between sentences in the English text, that is, the coherence mode. We exploit the improved VF2 subgraph matching algorithm to mine frequently occurring subgraph patterns in sentence semantic graphs to capture coherent patterns in English text. Finally, in the coherence analysis of English text, we use a large number of English texts with good coherence to train to generate our frequent subatlas. According to the frequent subgraph patterns that appear in the English text to be tested, the overall coherence quality of the English text to be tested is studied by combining their frequency and the semantic value of the subgraphs. Comparative experiments are carried out from the text aspect to prove the effectiveness of the adaptive mechanism proposed in this paper in optimizing the neural network. The experimental results show that the algorithm has achieved satisfactory results in terms of classification and loss value on the text data set. Our model performs well in the coherence analysis of English texts.

The article "Application of Adaptive Neural Network Algorithm Model in English Text Analysis" was retracted in 2023. Reasons: signs of a paper mill; suspected computer-generated content; unreliable results or conclusions; concerns about the data.

## Figures and Tables

**Figure 1:** The overall structure of the encoder-decoder of the automatic syntax error correction model.

**Figure 2:** Description of the casual mask method in transformer.

**Figure 3:** Test accuracy with and without dropout: (a) test accuracy using dropout and (b) test accuracy without dropout.

**Figure 4:** The number of frequent subgraphs in different test texts.

**Figure 5:** Experiments on incoherent sentence extraction under different thresholds.

**Figure 6:** Experimental results of incoherent sentence extraction under different numbers of English compositions.

**Figure 7:** The real-time performance of sentence sorting for different models.

**Figure 8:** Comparison of English composition coherence quality scores.

## Data Availability

The data used to support the findings of this study are available from the corresponding author upon request.
